The article "Deciphering the Urinary Microbiota Repertoire by Culturomics Reveals Mostly Anaerobic Bacteria From the Gut" was retracted in 2025. Reasons: unreliable results or conclusions; lack of ethics approval or compliance.

# Deciphering the Urinary Microbiota Repertoire by Culturomics Reveals Mostly Anaerobic Bacteria From the Gut

**DOI:** 10.3389/fmicb.2020.513305

**Published:** 2020-10-16

**Authors:** Grégory Dubourg, Aurélie Morand, Fatima Mekhalif, Raphael Godefroy, Alice Corthier, Abdourahamane Yacouba, Ami Diakite, Florent Cornu, Marina Cresci, Samy Brahimi, Aurélia Caputo, Eric Lechevallier, Michel Tsimaratos, Valérie Moal, Jean-Christophe Lagier, Didier Raoult

**Affiliations:** ^1^IRD, AP-HM, Microbes, Evolution, Phylogeny and Infection (MEPHI), IHU Méditerranée Infection, Aix-Marseille University, Marseille, France; ^2^Pédiatrie Spécialisée et Médecine Infantile, Hôpital de la Timone, AP-HM, Marseille, France; ^3^Fondation Méditerranée Infection, Marseille, France; ^4^Department of Urology and Renal Transplantation, La Conception University Hospital, AP-HM, Aix-Marseille University, Marseille, France; ^5^Pédiatrie Multidisciplinaire, Hôpital de la Timone, AP-HM, Marseille, France; ^6^Centre de Nephrologie et Transplantation Rénale, Hôpital de la Conception, Aix-Marseille University, Marseille, France

**Keywords:** urine, microbiota, culturomics, bladder, culture

## Abstract

Human urine was considered sterile for a long time. However, 416 species have been previously cultured, including only 40 anaerobic species. Here, we used culturomics, particularly those targeting anaerobes, to better understand the urinary microbiota. By testing 435 urine samples, we isolated 450 different bacterial species, including 256 never described in urine of which 18 were new species. Among the bacterial species identified, 161 were anaerobes (35%). This study increased the known urine repertoire by 39%. Among the 672 bacterial species isolated now at least once from urine microbiota, 431 (64.1%) were previously isolated from gut microbiota, while only 213 (31.7%) were previously isolated from vagina. These results suggest that many members of the microbiota in the urinary tract are in fact derived from the gut, and a paradigm shift is thus needed in our understanding.

## Introduction

The study of the urinary microbiota is recent and has been subjected to many biases. Indeed, since urine has been considered naturally sterile (Wolfe et al., 2012; Hilt et al., 2014) due to methodological biases, the techniques developed to detect bacteria of urinary origin have led to the consideration of only dominant bacteria from easily, rapidly, and aerobically cultured (Moroni et al., 1976; Bennett et al., 2014) urinary specimens. In addition, the higher frequency of urinary tract infections (UTIs) in women than in men has led to the consideration that the source of bladder colonization is genital due to the small size of the female urethra (Hooton, 2001). By analogy, this has led to the hypothesis that the bladder microbiota, apart from UTIs, is of vaginal origin, neglecting the fact that men also have UTIs (Wagenlehner et al., 2014) and a urinary microbiota. We have recently constituted a database of bacteria isolated from the urinary tract containing 416 cultured bacterial species (Morand et al., 2019) that were cultured before the present study. We have developed a high-throughput culture approach entitled culturomics that relies on the multiplication of culture conditions, thereby allowing to isolate bacteria that were considered as unculturable (Lagier et al., 2012) by multiplying culture conditions. This approach enabled a significant increase of repertoire of prokaryotes associated with human gut (Lagier et al., 2016) through the discovery of hundreds of new taxa. The aim of the present study was therefore to explore the urinary microbiota as we previously did for the gut microbiota (Lagier et al., 2016; Bilen et al., 2018) by using anaerobic culture techniques on urinary samples collected from men and women.

## Materials and Methods

### Ethics

Ethical approval was obtained for the UTI project under the number 2015-A00884-45. The ethics committee of the Institut Hospitalo-Universitaire (IHU) Méditerranée Infection validated the study under numbers 2016-001, 2016-010, 2016-011, and 2017-026-03. Regarding the inclusion of children, the study was explained to the parents, and a consent form was given to the parents.

### Study Design

This study was segmented in 13 different projects conducted over 5 years (Table 1). Urine was sampled in accordance with the relevant procedures for collecting samples dedicated to the microbiological diagnosis of UTIs (Supplementary Material). All the urine samples were quickly transported to the laboratory to be inoculated in culture media in the 6 h following the urine collection. All the samples were separated into three specimens: one for the routine microbiology laboratory, one dedicated to the culturomics analysis, and one aliquot of 1 mL was frozen at −80°C when a sufficient volume was available.

**TABLE 1:** Summary of the different projects included in this study.

Project	Year	No. of samples	No. of conditions used	No. of colonies tested	No. of species cultured
Children with urologic diseases	2015	11	11	10,212	96
Renal transplant 1st cohort	2015	70	3	3,787	110
Renal transplant/donors 2nd cohort	2016	65	8	5,400	139
Newborn	2017	31	8	7,152	124
UTI	2017	17	8	10,000	78
FMT	2018	11	4	7,104	74
Probiotics	2018	132	4	85,500	276
Renal transplant/donors 3rd cohort	2018	10	8	3,200	123
Renal transplant/donors 4th cohort	2019	68	8	2,868	112
Suspected bladder cancer	2019	20	11	8,466	51

### Culturomics

A total of 26 different culture conditions were designed for this purpose (Supplementary Data Sheet 1). However, depending on the volume of urine collected and the purpose of each project (Lagier et al., 2019), the number of conditions per project ranged between three and 11 culture conditions (see Supplementary Methods). A volume of at least 100 μL was inoculated for each condition. Inoculation onto Columbia with 5% sheep blood agar in aerobic and anaerobic atmospheres was systematically performed while plating on R-medium (Dione et al., 2016) and pre-incubation in blood culture bottles were the following most used culture conditions (in 82% and 73% of the projects included, respectively). Identification of colonies was performed using Matrix Assisted Laser Desorption Ionization-Time of Flight Mass Spectrometry (MALDI-TOF MS) (Seng et al., 2009). Isolates with an identification score > 2 with a unique hit were considered as accurately identified. In other cases (i.e., low score or multiple hit with same score), 16S rRNA gene sequencing was carried out to achieve final identification (Morel et al., 2015) (Supplementary Material). A new species was defined by a 16S rRNA gene sequence homology below 98.65% with that of the phylogenetically closest neighbor validated in standing nomenclature (Stackebrandt, 2006; Meier-Kolthoff et al., 2013). The genomes of these taxa were then sequenced as previously described (Alou et al., 2018).

### Microbiota Analysis by 16S rRNA Gene Analysis

We performed the 16S rRNA gene sequencing on 378 urinary specimens by targeting the V3-V4 regions using an Illumina MiSeq platform (see Supplementary Methods). Taxonomic assignment was performed using a custom database containing 76,368 sequences to perform our analysis and including sequences of species isolated as a part of culturomics studies or from the routine diagnostic laboratory (Supplementary Methods) as previously described (Diakite et al., 2019). To estimate the percentage of uncultured bacteria that may remain to be discovered we have pooled the sequences obtained from the 378 urinary samples and then compared the operational taxonomic unit (OTU) detected with the species cultured in this study. When an OTU comprises several species clustered with the same homology, we considered that the OTU was also detected by culturomics if at least one species belonging to this cluster was isolated.

### Graphical Representation and Statistical Analysis

Statistical tests were performed using GraphPad Prism v7.0 (La Jolla, CA, United States), while Venn diagrams were generated using InteractiVenn (Heberle et al., 2015).

## Results

### Expansion of the Urinary Repertoire of Microbes

Overall, by analyzing 143,689 colonies, we cultured a total of 435 urine specimens from 279 patients and identified 457 microorganisms of which seven were fungi (*Candida parapsilosis, Candida tropicalis, Candida krusei, Candida albicans, Candida glabrata*, *Candida kefyr* and *Trichosporon inkin*). Among the 450 bacteria cultured, 194 were already known from a previously established repertoire of bacteria cultured from the urinary tract and 256 bacterial species had not previously been identified from urine specimens (Figure 1). Of these, 182 were previously identified from humans. Thanks to the shared databases between different MALDI-TOF devices used in the laboratory, 45 species that were previously discovered as a part of culturomics studies were identified in urine specimens (Supplementary Table 1). Most of these taxa were first isolated from the human gut (30/45, 66.7%), 14 were isolated from vaginal specimens and one from sputum samples. Of the 29 species that were not previously detected in humans, 11 were previously recognized taxa. Among the main discoveries, the present study was able to isolate 18 different new species and genera (Cresci et al., 2016; Morand et al., 2016a,b,c; Brahimi et al., 2017a,b,c,d; Niang et al., 2019a,b; Yimagou et al., 2019) (Table 2). Of these, seven (39%) were detected in several projects. In addition, *Actinomyces urinae* was cultured in four different projects, highlighting the probable high prevalence of the species in the urinary tract. Due to these culturomics studies, the number of bacteria known in the urinary tract is now 672, thereby extending the prokaryotic urinary repertoire by 37%. When focusing on these 256 bacteria added to the repertoire, Firmicutes were most represented (130 species, 50.7%) followed by Actinobacteria (65 species, 25%). Species from phyla rarely encountered in urine were also added, such as Fusobacteria (i.e., *Fusobacterium naviforme and F. necrophorum*). Interestingly, we cultured two species from the Synergistetes phylum that has rarely been found by culture approach. Indeed, *Pyramidobacter piscolens* was previously isolated from the oral cavity and the gut microbiota (Downes et al., 2009), and *Jonquetella anthropi* was initially recovered from clinical specimens (Jumas-Bilak et al., 2007). The family Peptoniphilaceae contributed to extending the repertoire the most because it represents 8% of the species added. This family contains mainly anaerobes; therefore, we looked at the tolerance to oxygen of the bacteria recovered in this study. Among the 256 additional species, 130 were strict anaerobes (50.7%). In the previously established repertoire (Morand et al., 2019), only 9.4% of the cultivated species were anaerobes, the same ratio being 35% when considering only the present study, highlighting that anaerobes were so far ignored from the urinary tract.

**FIGURE 1:** Evolution over time of the urinary repertoire according to culturomics studies. The bacterial species are represented in five categories: Known in urines, prokaryotes isolated by other laboratories but not by culturomics; identified in urines by culturomics, taxa recovered by culturomics studies and already known to belong to the bacterial urinary repertoire; new species culturomics, new taxa discovered as a part of other culturomics studies; unknown in humans, prokaryotes first isolated in humans; and new species culturomics urines, species isolated from urinary tract as a part of this study.

**TABLE 2:** Main characteristics of the 18 new species isolated as a part of this study including strain collection deposit number, 16S rRNA sequence accession number, genome accession number (when available), and culture conditions required for primo-isolation and reference (when available).

Species	Strain number	16S rRNA sequence accession number	Genome accession number	Culture condition used for the first isolation	References
*Actinomyces urinae*	P2225	LN870295	FPKP01000000	Pre-incubation in anaerobic blood culture bottle during 10 days at 37°C and subculture onto Columbia agar + 5% sheep blood in anaerobic conditions	Morand et al., 2016c
*Actinotignum timonense*	P2803	LT598555	FTLO0000000	Direct seeding on a 5% sheep blood Columbia agar medium incubated at 37°C in aerobic atmosphere during 7 days	Brahimi et al., 2017b
*Anaerococcus urinomassiliensis*	P2143	LN898272	FQRX01000000	Pre-incubation during 10 days in an anaerobic blood culture vial supplemented with rumen fluid and subculture at 37°C on 5% sheep blood–Columbia agar	Morand et al., 2016b
*Arcanobacterium urinimassiliense*	P3248	LT598574	FPJH00000000	Pre-incubation in an anaerobic blood culture bottle supplemented with rumen and blood during 30 days followed by a 3 days subculture on R-medium during 3 days	Diop et al., 2017
*Bacteroides transplantocaccae*	P8575	LR745843	PRJEB36169	Direct seeding on a 5% sheep blood Columbia agar medium incubated at 37°C in aerobic atmosphere during 2 days	Unpublished
*Corynebacterium lascolaense*	P2174	LN881612	FMSX00000000	Direct seeding onto 5% sheep’s blood–enriched Columbia agar at 37°C in aerobic atmosphere	Unpublished
*Corynebacterium phoceense*	P1905	LN849777	FLTI01000001	Direct seeding onto 5% sheep’s blood–enriched Columbia agar at 37°C in aerobic atmosphere	Cresci et al., 2016
*Corynebacterium urinale*	P3884	LR135787	NA	Direct seeding on a 5% sheep blood Columbia agar medium incubated at 37°C in aerobic atmosphere during 1 day	Unpublished
*Corynebacterium urinapleomorphum*	P2799	LT576404	FTLL00000000	Direct seeding onto 5% sheep’s blood–antioxidant agar homemade R-medium in anaerobic atmosphere at 37°C during 3 days	Niang et al., 2019b
*Lachnoclostridium phocaeense*	P3177	LT598581	LT635479	Pre-incubation in an anaerobic blood culture bottle rumen fluid and sheep’s blood during 96 hours and subculture on 5% sheep’s blood–enriched Columbia agar after 5 days at 37°C under anaerobic atmosphere	Brahimi et al., 2017c
*Lachnoclostridium urinimassiliense*	P2804	LT576406	NA	Pre-incubation in an anaerobic blood culture bottle supplemented with rumen and sheep’s blood during 96 hours and subculture on 5% sheep’s blood Columbia agar after 3 days at 37°C under anaerobic atmosphere	Brahimi et al., 2017c
*Ndongobacter massiliensis*	P3170	LT598585	LT635480	Pre-incubation in an anaerobic blood-culture bottle enriched with rumen during 10 days and subculture on 5% sheep blood Columbia agar medium after 3 days of incubation at 37°C in an anaerobic atmosphere	Brahimi et al., 2017d
*Olsenella urininfantis*	P3197	LT598594	FTLR00000000	Pre-incubation during 30 days in an anaerobic blood culture supplemented with rumen fluid and sheep blood subcultured on 5% sheep blood-enriched Columbia agar at 37°C in anaerobic atmosphere during 72 h	Morand et al., 2016a
*Pelistega massiliensis*	P2015	LN881604	FMSW00000000	NA	Unpublished
*Peptoniphilus urinimassiliensis*	P3195	LT598577	FTPC00000000	Direct seeding onto 5% sheep blood Columbia agar medium 37°C in an anaerobic atmosphere during 4 days	Brahimi et al., 2017d
*Streptococcus transplantocaccae*	P9010	LR792269	CADEHI010000000	Direct seeding on a 5% sheep blood Columbia agar medium incubated at 37°C in aerobic atmosphere during 2 days	Unpublished
*Urinicoccus massiliensis*	P1992	LN881616	FPLH00000000	Pre-incubation in a blood culture vial supplemented with rumen fluid in anaerobic conditions at 37°C during 10 days and subcultured onto 5% sheep blood agar in anaerobic atmosphere	Yimagou et al., 2019
*Varibaculum massiliense*	P2802	LT576396	FNWI00000000	Direct seeding on a 5% sheep’s blood Columbia agar for 7 days at 37°C in anaerobic atmosphere	Niang et al., 2019a

*NA: not available.*

### Presence of Uropathogens in Urinary Specimen

We looked at the prevalence of uropathogens (see Supplementary Material, Section 4.1) in a subset of 406 urinary samples with corresponding gender information. We found a non-significant difference regarding the presence of at least one uropathogen between male (107/195, 54.8%) and female (129/212, 60.8%) specimens (Fischer exact test, *p* = 0.12) (Figure 2A). Nevertheless, the number of uropathogens cultured per urinary sample was different between males and females (Mann and Whitney test, *p* = 0.032) (Figure 2B), and *E. coli* was more frequently found in specimens from women (58/212, 37.9%) than in those from men (36/195, 18.5%) (Fischer’s exact test *p* = 0.03) (Figure 2C).

**FIGURE 2:** Number of specimens for which at least one uropathogen **(A)** and *E. coli* **(C)** were recovered by culture in this study, respectively, among male and female patients. **(B)** highlights the median number of uropathogens cultured per sample among men and women. *p < 0.05.

### Putative Source of the Microbes Cultured

We attempted to identify the potential source of the microbes inhabiting the urinary tract by comparing the current updated repertoire of bacteria cultured from urine (Morand et al., 2019 and this study combined) with those established from the gut (Lagier et al., 2016), the respiratory tract (Fonkou et al., 2018), and the vagina (Diop et al., 2019). Strikingly, the majority of the 672 species (i.e., 64.1%) cultured from urine were shared with the human gut repertoire (Figure 3), while less than half were shared with vaginal and respiratory/oral cavity microbiomes (i.e., 31.7% and 40%, respectively) (Supplementary Table 2). We also looked at the 10 most prevalent bacteria retrieved from urine specimens in clinical microbiology laboratories over a five-year period. Compared to males, females were found to have more *S. agalactiae* and *Staphylococcus saprophyticus* (Table 3). In addition, six and seven bacteria from this ranking list from male and female specimens, respectively, are common residents of the digestive tract. Finally, when comparing the species recovered from male and female subjects in this study, a substantial proportion (i.e., 48%) was found in both groups (Supplementary Table 3).

**FIGURE 3:** Venn diagram showing the shared cultured species between the human urinary tract (this study and Morand et al., 2019), the human gut (Lagier et al., 2016), the human respiratory tract/oral cavity (Fonkou et al., 2018), and the human vagina (Diop et al., 2019).

**TABLE 3:** List of the 10 most prevalent bacteria retrieved from urinary samples analyzed in the clinical microbiology laboratory (IHU Mediterranée Infection) from both male and female specimens.

Species	No.	Frequency by gender
**Female subjects**		
*Escherichia coli*	23,950	57.00%
*Klebsiella pneumoniae*	4,308	10.30%
*Enterococcus faecalis*	2,425	5.80%
*Proteus mirabilis*	1,572	3.70%
*Streptococcus agalactiae*	1,321	3.10%
*Pseudomonas aeruginosa*	1,171	2.80%
*Staphylococcus saprophyticus*	828	2.00%
*Enterobacter cloacae*	735	1.80%
*Enterococcus faecium*	528	1.30%
*Staphylococcus epidermidis*	495	1.20%
**Male subjects**		
*Escherichia coli*	8,218	34.00%
*Enterococcus faecalis*	2,945	12.20%
*Klebsiella pneumonia*	2,735	11.30%
*Pseudomonas aeruginosa*	1,632	6.80%
*Enterobacter cloacae*	1,119	4.60%
*Proteus mirabilis*	1,025	4.20%
*Staphylococcus epidermidis*	910	3.80%
*Staphylococcus aureus*	721	3.00%
*Klebsiella oxytoca*	512	2.10%
*Citrobacter koseri*	461	1.90%

*Extracted data extracted specimens collected from February 10, 2014 to June 8, 2019. A total of 75,707 bacterial identifications were performed, accounting for 66,141 positive samples. Data were de-replicated per both hospitalization stay and microbe.*

### Comparison of Urinary Microbiotas by Culturomics and 16S rRNA Gene Analysis

The 16S rRNA gene analysis applied on the 378 urinary generated a total of 16,937,127 reads accurately assigned to bacteria accounting for 3,484 OTU. The 1,305 OTU assigned to known species represented 94.3% of the total number of reads (i.e., 15,942,967). We found that 375 of these 1,305 OTU (28.7%) overlapped with species isolated by culture. However, this represents 62.2% (i.e., 10,538,786 reads) of the number of reads assigned to known species. On the other hand, 165 of the 450 cultured bacteria (37%) were not detected by sequencing.

We performed the same analysis by excluding OTU representing less than 0.001% of total sequences. As a result, 1,062 OTU assigned to bacteria were kept and accounted for 16,782,244 reads. The 674 OTU assigned to known species represented 94.7% of the total number of reads (i.e., 15,896,084 reads). We found that 258 of these 674 OTU (38.2%) overlapped with species isolated by culture that represents 66.2% (i.e., 10,530,485 reads) of the number of reads assigned to known species. Interestingly, 170 of the cultured bacteria were missed by 16S rRNA gene sequencing, highlighting that 25 additional bacterial species found in culture are not detected anymore following the exclusion of rare OTU. Of these species, four are new taxa previously discovered by culturomics, and one is a new species isolated as a part of this study (i.e., *Urinacoccus massiliensis*). These results suggest that removing low abundances OTU may lead to underestimate bacterial diversity from sequencing datasets (Supplementary Table 4).

## Discussion

In this exploratory study, we report the culture of 457 microorganisms from urinary specimens by a culturomics approach, of which 450 were bacteria. The current work enriches the current human microbiota repertoire of 39% because the number of bacteria cultured from the human urinary microbiota has reached 672 bacterial species thanks to this study. In this study, 66% of the sequences generated by whole microbiota analysis were from cultured bacteria while a substantial number of the bacteria isolated in this work (i.e., 166 bacterial species, 37%) were not detected by molecular approaches.

The current work shows that men have a microbiota as diverse as women (Supplementary Table 3) and, as a result, raises the question about the exclusive vaginal origin of the female bladder microbiota, even if some microorganisms are found in common in the vagina and urine. The source of vaginal bacteria can be both urinary and fecal in origin. Anatomically, it seems more directly related to a urinary source than to a fecal source, but strikingly, 64.1% of the 672 species that have been found at least once in urine specimen were already cultured from human gut (Figure 3 and Supplementary Table 2). Moreover, out of the 45 species cultured and that were formerly discovered as a part of culturomics studies, 30 (67%) were initially isolated from fecal specimen (Supplementary Table 1). We also noticed that the urinary microbiota overlapped more with the respiratory/oral microbiotas than the vaginal microbiota (i.e., 40% and 32%, respectively). This is probably due to the high contribution of the gut microbiota that represents 76% (209/276) of the shared species. In addition, we found bacteria that have not been identified until now because they are strict anaerobes. The fact that 49.3% of the anaerobic species identified in this study were detected in at least two subprojects highlights that they are in fact commensal of the urinary tract (Supplementary Table 1). There is, however, no systematic protocol dedicated to their culture because their impact on UTIs was considered negligible. This is exemplified by a recent study suggesting a shared microbiota between the vagina and bladder by culturing 149 bacterial strains, of which several strains cultivated from the two sites displayed a high level of similarity (Thomas-White et al., 2018). Indeed, the authors did not perform extensive anaerobic cultures because the media were only kept for 48 h, which can lead to erroneous conclusions. Again, the fact that studies of the urinary microbiota were deduced from UTIs led to a poor choice of strategy to discover the real microbiota. This was recently illustrated by the fact that *Methanobrevibacter smithii*, which is a very strict anaerobic Archae, was found in urine by two teams (Grine et al., 2019).

We assume that a substantial fraction of the specimen included in this study was mostly collected by urination and that potential urethral contamination could exist and that our findings have to be confirmed from catheterized urines. Nevertheless, the specimens were collected in accordance with the relevant procedures for collecting samples for microbiological purposes. Our study nevertheless constitutes a paradigm shift demonstrating that the origin of the urinary microbiota is the digestive tract. As a matter of fact, gut microbiota contributing to the diversity of prokaryotes inhabiting the urinary tract was suggested by a recent study highlighting the reduction in the recurrence of UTIs following fecal microbiota transplantation (FMT)(Staley et al., 2017; Tariq et al., 2017). It has also been recently suggested that the composition of the intestinal microbiota could impact the occurrence of UTI in children (Paalanne et al., 2018). These data suggest that UTI are in fact the consequences of ecosystem disruptions and that uropathogens could be acquired from the environment, particularly from animals (Jakobsen et al., 2010; Giufre et al., 2012; Maluta et al., 2014; Mellata et al., 2018). Supporting this, a systematic review demonstrated that half of the bacteria cultured from human milk have a probable digestive source (Togo et al., 2018). As a subproject of this study, we recently demonstrated the direct passage of *Lactobacillus* species directly through urine following yogurt ingestion (Lagier et al., 2019). Recent studies dedicated to the influence of urinary microbiota on bladder cancer nevertheless incriminate bacteria mostly derived from the gut (Wu et al., 2018; Bi et al., 2019). It therefore appears that tissue microbiota considered, until recently, sterile are in fact colonized by bacteria that are often fastidious and anaerobic and that have passed through the digestive tract. Further works, including those related to the subprojects included in this study, will shed light on the contributing role of these urinary commensals in health and disease.

## Data Availability Statement

The datasets generated for this study can be found in the NCBI under Run/Assembly accession numbers ranging from ERR3999831 to ERR4000209.

## Ethics Statement

The studies involving human participants were reviewed and approved by the Institut Hospitalo-Universitaire (IHU) Méditerranée Infection Ethics Committee, and the committee validated the study under numbers 2015-A00884-45, 2016-001, 2016-010, 2016-011, and 2017-026-03.

## Author Contributions

DR conceived and designed the experiments. VM, MT, and EL actively participated in the specimen collection and the study design. AM, FM, RG, ACo, AY, AD, FC, MC, and SB performed the culturomics experiments. ACa performed the bioinformatics analysis. GD, AM, J-CL, and DR analyzed the data. GD, AM, J-CL, and DR wrote the manuscript. All authors read and approved the final manuscript.

## Conflict of Interest

DR is a co-inventor of a patent on the culture of anaerobic bacteria (CAS 28-FR1757574). The remaining authors declare that the research was conducted in the absence of any commercial or financial relationships that could be construed as a potential conflict of interest.
